The article "Causal associations of gut microbiota and metabolites on sepsis: a two-sample Mendelian randomization study" was published in 2023. Journal: Front Immunol.

# Causal associations of gut microbiota and metabolites on sepsis: a two-sample Mendelian randomization study

**DOI:** 10.3389/fimmu.2023.1190230

**Published:** 2023-09-14

**Authors:** Jian Zhao, Xin Pan, Di Hao, Yi Zhao, Yuanzhuo Chen, Shuqin Zhou, Hu Peng, Yugang Zhuang

**Affiliations:** ^1^ Department of Emergency, Shanghai Tenth People’s Hospital, Tongji University School of Medicine, Shanghai, China; ^2^ Department of Gerontology, Shanghai Tenth People’s Hospital, Tongji University School of Medicine, Shanghai, China

**Keywords:** sepsis, gut microbiota, gut metabolites, Mendelian randomization, causal associations

## Abstract

**Background:**

Sepsis stands as a dire medical condition, arising when the body’s immune response to infection spirals into overdrive, paving the way for potential organ damage and potential mortality. With intestinal flora’s known impact on sepsis but a dearth of comprehensive data, our study embarked on a two-sample Mendelian randomization analysis to probe the causal link between gut microbiota and their metabolites with severe sepsis patients who succumbed within a 28-day span.

**Methods:**

Leveraging data from Genome-wide association study (GWAS) and combining it with data from 2,076 European descendants in the Framingham Heart Study, single-nucleotide polymorphisms (SNPs) were employed as Instrumental Variables (IVs) to discern gene loci affiliated with metabolites. GWAS summary statistics for sepsis were extracted from the UK Biobank consortium.

**Results:**

In this extensive exploration, 93 distinct genome-wide significant SNPs correlated with gut microbial metabolites and specific bacterial traits were identified for IVs construction. Notably, a substantial link between Coprococcus2 and both the incidence (OR of 0.80, 95% CI: 0.68-0.94, *P*=0.007) and the 28-day mortality rate (OR 0.48, 95% CI: 0.27-0.85, *P*=0.013) of sepsis was observed. The metabolite α-hydroxybutyrate displayed a marked association with sepsis onset (OR=1.08, 95% CI: 1.02-1.15, *P*=0.006) and its 28-day mortality rate (OR=1.17, 95% CI: 1.01-1.36, *P*=0.029).

**Conclusion:**

This research unveils the intricate interplay between the gut microbial consortium, especially the genus Coprococcus, and the metabolite α-hydroxybutyrate in the milieu of sepsis. The findings illuminate the pivotal role of intestinal microbiota and their metabolites in sepsis’ pathogenesis, offering fresh insights for future research and hinting at novel strategies for sepsis’ diagnosis, therapeutic interventions, and prognostic assessments.

## Introduction

Sepsis is a critical medical condition arising when the body’s immune response to an infection becomes overactive, leading to potential organ damage and even death (1). This condition is a pressing public health issue, impacting approximately 1.7 million individuals annually in the USA alone, with a fatality rate reaching nearly 50% (2, 3). Although its prevalence and severe consequences are alarming, treatment options for sepsis remain limited, primarily revolving around antibiotics and supportive therapies for many years.

The article "Causal associations of gut microbiota and metabolites on sepsis: a two-sample Mendelian randomization study" was published in 2023. Journal: Front Immunol.

In the annals of medicine, the intestines were once considered the primary nexus for sepsis and multi-organ dysfunction syndromes (4, 5). However, as our comprehension of the intestine’s role in sepsis has deepened, this perspective has unfurled its intricate nuances.Utilizing cutting-edge technologies such as 16S rRNA and whole-genome sequencing, the pivotal role of the microbial community in the pathogenesis of sepsis has been illuminated (6). Sepsis can profoundly disrupt the microbial equilibrium of the gut (4, 5). For instance, in critically ill patients, beneficial bacteria like Faecalibacterium spp and Prevotella spp, known producers of short chain fatty acids(SCFAs), are notably diminished (7). In contrast, certain pathogenic and antibiotic-resistant bacteria such as Clostridia spp and Enterococcae spp proliferate significantly within septic patients (8).This microbial imbalance not only reshapes the bacterial community but also impinges on immune responses. For example, segmented filamentous bacteria can stimulate B cells to produce Immunoglobulin A, while concurrently increasing the count of inflammatory Th17 cells (9). Additionally, commensal bacteria, by breaking down polysaccharides into SCFAs, not only fortify the intestinal protective barrier but also activate regulatory T cells, thus influencing the overarching immune milieu (9).

However, due to methodological disparities and varied outcome metrics, research in this domain is replete with challenges. Moreover, scant data from studies with limited samples substantiate the nexus between sepsis, intestinal flora, and associated metabolites. To bridge these lacunae, we embarked on a two-sample Mendelian randomization analysis to elucidate the causal linkage between gut microbiota and those severe sepsis patients who succumbed within a 28-day window. Mendelian randomization (MR) harnesses genetic variants as Instrumental Variables (IVs), simulating a randomized controlled trial and thereby attenuating biases and inaccuracies, fortifying the causal inference between exposure and aftermath (10, 11). Our endeavor aspires to enrich our grasp of the processes whereby the gut biome catalyzes ailments and foster the genesis of bespoke therapies anchored in microbiome modulations.

The article "Causal associations of gut microbiota and metabolites on sepsis: a two-sample Mendelian randomization study" was published in 2023. Journal: Front Immunol.

To the best of our discernment, ours stands as the inaugural exploration delving into the causal nexus between gut microbiota, metabolites, and sepsis in the departed. Our revelations intimate a plausible causative interconnection between gut microbiota, their metabolites, and severe sepsis, underscoring the imperative for continued scrutiny and bespoke microbiome stratagems to enhance the prognosis of sepsis.

## Materials and methods

### Study design

The MR study was predicated on three cardinal postulations, delineated in **Figure 1**. The first assumption is that genetic instrumental variants exhibit a robust association with the exposure. The second assumption is that these genetic instrumental variants remain unaffiliated with any conceivable confounders. The third assumption is that such genetic instrumental variants correlate with the outcome solely through the conduit of exposure (12, 13).

**Figure 1:** Directed acyclic graphs for the classical Mendelian randomization designs. The arrows denote causal relations between two variables, pointing from the cause to the effect. The causal pathway is blocked if”X”is placed in the arrowed line. MR, Mendelian randomization.

### Data sources

The study gathered data on gut microbial metabolites, including α-hydroxybutyrate,β-aminoisobutyric acid, Thyroxine,Phosphodiesterase,Xanthosine through summary data from Genome-wide association study (GWAS). The data was collected from 2,076 participants of European descent in the Framingham Heart Study. To identify gene loci associated with these metabolites, the study used single-nucleotide polymorphisms(SNPs) that met suggestive genome-wide significance thresholds, with a *P* value of less than 5 × 10^-5^ as IVs (14).

The gut microbiota summary statistics was extracted from an extensive genetic survey encompassing 18,340 participants spanning 24 diverse cohorts. This investigation catalogued 211taxa, subdivided into 131genera, 35 families, 20orders, 16classes, and 9phyla. Organisms such as Coprococcus2, Ruminococcaceae UCG011, and Lachnospiraceae FCS020 group were scrutinized, with SNPs brandishing *P* values beneath 5 × 10^-5^ earmarked as IVs (15).

The GWAS summary statistics for sepsis were sourced from the data released by the UK Biobank consortium. Additionally, these statistics can be accessed through the IEU Open GWAS website, under the identifiers ieu-b-4982 (for sepsis) and ieu-b-4981 (for 28-day mortality). The dataset comprises a sample size of 431,365, of which 1,380 individuals were diagnosed with sepsis and 347 experienced mortality within a 28-day period.

### Instrumental variable selection

The following selection criteria were used to choose the Instrumental Variables (1): single nucleotide polymorphisms associated with each genus at the locus-wide significance threshold (*P* < 1× 10^-5^) were selected as potential IVs; (2) 1000 Genomes project European samples data were used as the reference panel to calculate the linkage disequilibrium between the SNPs, and among those SNPs that had r^2^ < 0.001 (clumping window size=10,000 kb), only the SNPs with the lowest *P* values were retained; (3) SNPs with minor allele frequency ≤ 0.01 were removed; and (4) when palindromic SNPs existed, the forward strand alleles were inferred using allele frequency information (16).

The article "Causal associations of gut microbiota and metabolites on sepsis: a two-sample Mendelian randomization study" was published in 2023. Journal: Front Immunol.

The strength of IVs was assessed by calculating the F-statistic using the formula F = R^2^× (N−1−K) (1−R^2^) × K, where R^2^ represents the proportion of variance in the exposure explained by the genetic variants, N represents sample size, and K represents the number of instruments the corresponding F-statistic was >10, it was considered that there was no significant weak instrumental bias (17).

### Mendelian randomization analysis

We used five methods for performing MR analysis, including the inverse variance weighted (IVW), multiplicative random effects (MR-Egger), weighted median, simple mode, and weighted mode. IVW, the most commonly used and efficient method, was selected as the primary analysis for this study, as it provides an estimate with the highest power, relying on the assumption that all SNPs are valid instrumental variables. When the assumption of no pleiotropy is violated, MR-Egger provides a more robust alternative. The weighted median, simple mode, and weighted mode each have their respective advantages and limitations and can be useful depending on the specific research question and available data. To validate the stability of our results, we also performed supplementary analyses using these three methods (18–20).

We conducted sensitivity analyses to assess the robustness of our findings, including two methods for detecting and addressing horizontal pleiotropy: MR-Egger regression and MR-PRESSO (21). Additionally, we used Cochran’s Q test to evaluate heterogeneity between SNPs associated with each microbial taxon (22). Lastly, we conducted a leave-one-out sensitivity analysis to evaluate the influence of individual SNPs on the overall estimates.

All MR analyses were performed in R (version 4.1.2) using R package TwoSampleMR and MRPRESSO (23).

## Result

### Participants and genetic instrumental variables in relation to gut microbiota and metabolites

In this comprehensive study, we identified 93 distinct genome-wide significant SNPs intricately linked with gut microbial metabolites and distinct bacterial attributes, which were harnessed for IVs construction. This includes 8 associated with Coprococcus2, 11 with Dialister, 8 with Ruminococcaceae UCG011, 11 with Coprococcus1, 12 with Lachnospiraceae FCS020 group, 8 with Ruminococcus torques group, 9 with Sellimonas, 5 with Terrisporobacter, 9 with Victivallis, 5 with α-hydroxybutyrate, 4 with cystine, 19 with β-aminoisobutyric acid, 6 with Thyroxine, 8 with phosphodiesterase, and 8 with Xanthosine. A robust F-statistic exceeding 20 suggests that this study is resistant to weak IVs bias.

The article "Causal associations of gut microbiota and metabolites on sepsis: a two-sample Mendelian randomization study" was published in 2023. Journal: Front Immunol.

### Mendelian randomization analysis of gut microbiota and sepsis

Upon thorough evaluation of multiple MR techniques, a notable correlation emerges between Coprococcus2 and both the incidence and 28-day mortality rate of sepsis, **Figure 2**. Specifically, IVW results delineate a significant inverse relation between Coprococcus2 and sepsis onset, with an OR of 0.80 (95% CI: 0.68-0.94, *P*=0.007), while for the 28-day mortality rate, the OR is 0.48 (95% CI: 0.27-0.85, *P*=0.013). Beyond Coprococcus2, there are conspicuous links with Dialister (OR=0.84, 95% CI: 0.74-0.96, *P*=0.016) and Ruminococcaceae UCG011 (OR=1.10, 95% CI: 1.01-1.20, *P*=0.024). For 28-day mortality, entities like Lachnospiraceae FCS020 group (OR=0.70, 95% CI: 0.51-0.95, *P*=0.023) and Ruminococcus torques group (OR=1.53, 95% CI: 1.00-2.34, *P*=0.049) manifest significant influence. Techniques including MR-egger, Weighted median, Simple mode, and Weighted mode align in direction with the IVW method, reinforcing the robustness of our findings. *P* values for Pleiotropy and Heterogeneity predominantly exceed 0.05, indicating the absence of significant heterogeneity or pleiotropy issues.

**Figure 2:** Forest plot to visualize the causal effect of Gut microbiota on the risk of Sepsis by inverse variance weighted method.

### Mendelian randomization analysis of gut metabolites and sepsis

α-hydroxybutyrate exhibits a pronounced relationship with both sepsis onset (OR=1.08, 95% CI: 1.02-1.15, *P*=0.006) and its 28-day mortality rate (OR=1.17, 95% CI: 1.01-1.36, *P*=0.029), **Figure 3**. Regarding sepsis onset, significant associations are evident with Cystine (OR=0.92, 95% CI: 0.85-0.99, *P*=0.029), β-aminoisobutyric acid (OR=1.03, 95% CI: 1.00-1.06, *P*=0.031), and Thyroxine (OR=0.95, 95% CI: 0.91-0.99, *P*=0.046). In terms of the 28-day mortality rate, Phosphodiesterase (OR=1.13, 95% CI: 1.02-1.26, *P*=0.016) and Xanthosine (OR=1.16, 95% CI: 1.02-1.32, *P*=0.021) both convey significant relationships. The outcomes from the MR-egger, Weighted median, Simple mode, and Weighted mode techniques are congruent with the direction of the IVW method, further corroborating the integrity of the primary findings. The *P* values for Pleiotropy and Heterogeneity mostly surpass 0.05, suggesting that the analytical results are steadfast and free from substantial heterogeneity or pleiotropy concerns.

The article "Causal associations of gut microbiota and metabolites on sepsis: a two-sample Mendelian randomization study" was published in 2023. Journal: Front Immunol.

**Figure 3:** Forest plot to visualize the causal effect of Gut Metabolites on the risk of Sepsis 28-day morality by inverse variance weighted method.

## Discussion

This study utilized the Mendelian Randomization approach to delve deeply into the association between gut microbiota, their metabolites, and sepsis. We successfully identified 93 SNPs significantly associated with gut microbial metabolites and specific bacterial attributes, providing a robust instrumental variable for the Mendelian Randomization analysis. Among these findings, the microbial communities notably associated with the incidence and 28-day mortality rate of sepsis included Coprococcus2, Dialister, and Ruminococcaceae UCG011. Notably, Coprococcus2 demonstrated a significant inverse correlation with both the onset of sepsis and the 28-day mortality rate. For microbial metabolites, we observed that α-hydroxybutyrate had a pronounced association with both the onset of sepsis and its 28-day mortality rate. Additionally, cystine, β-aminoisobutyric acid, and Thyroxine were closely associated with the incidence of sepsis. Furthermore, various Mendelian Randomization techniques yielded results consistent with our primary findings, reinforcing the robustness of our conclusions.

For generations, the intestinal microbiome has orchestrated myriad homeostatic functions in the hale host, encompassing both immune modulation and fortification of the gut barrier. Contemporary findings have illuminated an intricate nexus between the gut microbiome and sepsis. Antecedent to the advent of sepsis, perturbations within the gut microbiome exacerbate septic susceptibilities through an array of avenues: fostering the proliferation of deleterious intestinal flora, predisposing the immune apparatus to heightened inflammatory cascades, and curtailing the synthesis of salubrious microbial derivatives like short-chain fatty acids. With the inception of sepsis, the ensuing derangement of the intestinal microbiome augments end-organ malaise and amplifies vulnerability. Our investigation has discerned that Coprococcus2 bears a significant inverse correlation with both the incidence of septicemia and the 28-day mortality rate, corroborating Lufang Che’s observation in animal trials where septic mice models exhibited a diminished abundance of the Coprococcus genus, subsequently manifesting poorer prognostic outcomes (24). Furthermore, Jieyang Yu’s research has noted a waning abundance of Coprococcus in patients afflicted with sepsis (25). The mechanisms through which Coprococcus potentially influences sepsis could encompass several facets. Historically, studies have posited that Coprococcus can modulate the production of cytokines IL-1β and IL-6, thereby orchestrating the inflammatory response during an infection (26). Concurrently, Coprococcus is recognized as one of the principal bacteria responsible for butyrate production; butyrate, deemed a salubrious short-chain fatty acid, is pivotal for the health and functionality of colonic epithelial cells (16). Additionally, our research has identified α-hydroxybutyrate as closely intertwined with sepsis, qualifying it as a risk determinant for sepsis and the subsequent 28-day mortality rate. Historical studies have attested to the association of α-hydroxybutyrate with a gamut of ailments including diabetes, insulin resistance, obesity, and heart failure (27, 28). In certain contexts, it is perceived as a nascent biomarker for hypoxia and/or mitochondrial dysfunction (29). Recent inquiries indicate that elevated levels of α-hydroxybutyrate may portend adverse outcomes in COVID-19 patients, seemingly underscoring its distinctive role amidst infections (30, 31).

The article "Causal associations of gut microbiota and metabolites on sepsis: a two-sample Mendelian randomization study" was published in 2023. Journal: Front Immunol.

Our study illuminates the pivotal role of the gut microbiota, notably the genus Coprococcus and its metabolite α-hydroxybutyrate, within the trajectory of sepsis. Biologically construed, this suggests that the equilibrium of intestinal microbial communities and their resultant metabolites can either directly or tangentially shape the host’s immune responses and escalate the peril of disease exacerbation. In practical applications, this proffers a rejuvenated perspective where therapeutic strategies might transcend mere targeting of the pathogens, potentially venturing into modulating the intestinal microbial milieu. Furthermore, our insights underscore the quintessence of considering the gut microbiota and its metabolites when diagnosing and prognosticating the course of sepsis.

We posit a potential mechanism centered on the regulatory role of the Coprococcus genus over the host’s inflammatory dynamics. A diminishing presence of this bacterial lineage might instigate an amplified reactivity to inflammatory stimuli within the host, potentially intensifying the severity of sepsis. Moreover, this genus is heralded as a chief progenitor of butyrate, an entity esteemed indispensable for the vitality and operationality of colonic epithelial cells. A surge in α-hydroxybutyrate might be inextricably linked to mitochondrial impairments and/or cellular hypoxia, both cardinal players in the genesis and trajectory of sepsis.

The intricacies of our exploration merit attention. Firstly, the array of SNPs amassed, predicated upon the genome-wide statistical significance threshold (5 × 10^-8^), was too scant for exhaustive scrutiny. As a consequence, we embraced the SNPs that met the locus-wide significance criterion (5 × 10^-5^). Secondly, whilst the lion’s share of the GWAS summary data was sourced from European cohorts, a mere fraction of the gut microbiome information hailed from other ethnic backgrounds, possibly introducing a tint of bias into our observations. Thirdly, due to the confines of the foundational dataset, our probe was delimited to the genus tier, sidestepping finer subdivisions like species or strains. Nonetheless, the application of advanced shotgun metagenomic sequencing techniques might shed light with greater precision and nuance. Lastly, while our analysis was predicated solely on publicly available GWAS data, procuring raw clinical datasets for a thorough clinical investigation might yield more compelling outcomes.

The article "Causal associations of gut microbiota and metabolites on sepsis: a two-sample Mendelian randomization study" was published in 2023. Journal: Front Immunol.

## Conclusion

This investigation unveils the intimate interplay between the gut microbial consortium, notably the genus Coprococcus, and the metabolite α-hydroxybutyrate in the context of sepsis. Our revelations underscore the pivotal role of intestinal microbiota and their metabolites within the pathogenetic fabric of sepsis, charting fresh avenues for ensuing research. Concurrently, our outcomes proffer novel stratagems and methodologies for the diagnosis, therapeutic intervention, and prognostic evaluation of sepsis.

## Data availability statement

The original contributions presented in the study are included in the article/supplementary materials. Further inquiries can be directed to the corresponding authors.

## Ethics statement

The manuscript presents research on animals that do not require ethical approval for their study. Written informed consent was obtained from the minor(s)’ legal guardian/next of kin for the publication of any potentially identifiable images or data included in this article.

## Author contributions

HP and YuZ contributed to conception and design of the study. JZ and XP complete the review of literature and wrote the first draft of the manuscript. DH and YiZ conducted data acquisition and performed the statistical analysis. YC and SZ performed manuscript revision. All authors contributed to the article and approved the submitted version.
